# A positive feedback loop consisting of C12orf59/NF-κB/CDH11 promotes gastric cancer invasion and metastasis

This article has been retracted.

**DOI:** 10.1186/s13046-019-1114-2

**Published:** 2019-04-15

**Authors:** Jia-Xing Zhang, Wei-Ling He, Zi-Hao Feng, Dong-Liang Chen, Ying Gao, Ying He, Kai Qin, Zhou-San Zheng, Cui Chen, Hui-Wen Weng, Miao Yun, Sheng Ye, Rui-Hua Xu, Dan Xie

**Affiliations:** 1 The State Key Laboratory of Oncology in South China, Sun Yat-Sen University Cancer Center, Collaborative Innovation Center for Cancer Medicine, No. 651, Dongfeng Road East, 510060 Guangzhou, Guangdong Province People’s Republic of China; 2 Department of Oncology, the First Affiliated Hospital, Sun Yat-Sen University, Guangzhou, 510080 Guangdong Province People’s Republic of China; 3 Department of Gastrointestinal Surgery, The First Affiliated Hospital, Sun Yat-Sen University, Guangzhou, 510080 Guangdong Province People’s Republic of China; 4 Department of Urology, the First Affiliated Hospital, Sun Yat-Sen University, Guangzhou, 510080 Guangdong Province People’s Republic of China; 5 Department of Extracorporeal Circulation, the First Affiliated Hospital, Sun Yat-Sen University, Guangzhou, 510080 Guangdong Province People’s Republic of China

**Keywords:** Gastric cancer, C12orf59, NF-κB, CDH11, Metastasis

## Abstract

**Background:**

Metastasis remains the main cause of cancer-related death for gastric cancer (GC) patients, but the mechanisms are poorly understood. Using The Cancer Genome Atlas (TCGA) data base and bioinformatics analyses, we identified C12orf59 might act as a potential oncogenic protein in GC.

**Methods:**

We investigate the expression pattern and clinical significance of C12orf59 in two independent cohorts of GC samples. In the training cohort, we used the X-tile program software to generate the optimal cutoff value for C12orf59 expression in order to classify patients accurately according to clinical outcome. In the validation cohort, this derived cutoff score was applied to exam the association of C12orf59 expression with survival outcome. A series of in vivo and in vitro assays were then performed to investigate the function of C12orf59 in GC.

**Results:**

C12orf59 was significantly upregulated, and associated with poor survival outcome in two cohorts of GC samples. Gain- and loss of- function studies demonstrated C12orf59 promotes GC cell invasive and metastatic capacity both in vitro and in vivo, and induces epithelial–mesenchymal transition and angiogenesis. Mechanically, C12orf59 exerts oncogenic functions by up-regulating CDH11 expression via NF-κB signaling. Interesting, CDH11 could in turn promote NF-κB bind to C12orf59’s promoter and form a positive feedback loop to sustain the metastatic ability of GC cells. Additionally, downregulation of miR-654-5p is another important mechanism for C12orf59 overexpression in GC.

**Conclusion:**

Our finding suggested the newly identified C12orf59/NF-κB/CDH11 feedback loop may represent a new strategy for GC treatment.

**Electronic supplementary material:**

The online version of this article (10.1186/s13046-019-1114-2) contains supplementary material, which is available to authorized users.

## Background

Gastric cancer (GC) is one of the leading causes of cancer-related deaths worldwide. Despite of advancement of the surgical technique and the development of novel drugs, the overall survival (OS) of patients with GC remains poor [1, 2]. The mains cause of death in GC patients is tumor metastasis, but the underlying molecular mechanisms responsible for the development of metastasis are still not fully understood [3–5]. Thus, it is crucial and necessary to elucidate the molecular mechanism underlying invasiveness and metastasis of GC to identify novel therapeutic targets and develop new modalities of treatment.

Loss of tumor suppressor gene and activation of oncogenes are central events in GC tumorigenesis, and may contribute to the future malignant potential of the tumor [6, 7]. Thus, we attempted to search for novel molecules that regulate GC development and progression. To investigate the dysregulated gene profile that involved in GC tumorigenesis, we systematically analyzed microarray data of paired of GC cancer and non-cancerous tissues in The Cancer Genome Atlas (TCGA) database. We found that, Chromosome 12 open reading frame 59(*C12orf59*), localized on Chromosome 12p13.2, was significantly up-regulated in cancerous tissues of GC samples (Additional file 1: Figure S1a). *C12orf59,* a newly identified gene in kidney, was predicted to encode transmembrane proteins and associated with the RNA-binding protein HuR [8, 9]. Currently, the expression pattern and potential role of C12orf59 in human cancer types is largely unknown. Only one study reported that decreased C12orf59 expression was correlated with poor prognosis and von Hippel-Lindau (VHL) mutation in human Renal cell carcinoma (RCC) [10]. The significant aberration of C12orf59 in GC promoted us to further explore its potential oncogenic role in GC pathogenesis, although the function of C12orf59 in this disease is largely unknown.

In this study, we found that overexpression of C12orf59 correlated with poor survival prognosis of GC patients, and promoted GC cell invasion and metastasis both in vitro and in vivo. Mechanically, C12orf59 induces GC cell epithelial–mesenchymal transition (EMT) and angiogenesis by up-regulating CDH11 gene expression via NF-κB signaling. More importantly, CDH11 could in turn promote NF-κB bind to C12orf59’s promoter and form a positive feedback loop to sustain the metastatic ability of GC cells.

## Methods

### Patients and specimen collection

Two independent cohorts of 302 formalin-fixed paraffin-embedded (FFPE) tumor tissues and adjacent normal tissues (ANTs) of GC samples were included in present study. The training cohort was collected from 170 GC patients who underwent surgical resection from Sun Yat-Sen University Cancer Center (SYSUCC), between January 2010 and December 2011. In parallel, we obtained another validation cohort that consisted of 132 GC samples from the First Affiliated Hospital of Sun Yat-sen University, between January 2007 and May 2009. The patients enrolled were diagnosed with stage I-III GC during surgery resection, and did not receive any treatment before their operation. The clinicopathologic characteristics of the patients in each cohort are summarized in Table 1.

**Table 1:** Association of C12orf59 expression with patient’s clinicopathological features in GC

Variables	Case	Training cohort		*P*-value	Case	Validation cohort		*P*-value
		Low expression	High expression			Low expression	High expression	
Age		102	68			79	53	
≤60^a^	100	65 (50.9%)	35 (49.1%)		78	51 (54.5%)	27 (45.5%)	
>60	70	37 (58.1%)	33 (41.9%)	0.112	54	28 (53.5%)	26 (46.5%)	0.119
Gender								
Male	109	64 (50.0%)	45 (50.0%)		88	51 (50.0%)	37 (50.0%)	
Female	61	38 (63.3%)	23 (36.7%)	0.648	44	28 (63.3%)	16 (36.7%)	0.53
Tumor grade								
G1	56	39 (42.1%)	17 (57.8%)		38	23 (65.8%)	15 (34.2%)	
G2 + 3	114	63 (61.7%)	51 (38.3%)	0.072	94	56 (46.7%)	38 (53.3%)	0.92
Tumor size(cm)								
≤ 5^b^	91	59 (51.0%)	32 (49.0%)		97	62 (53.1%)	35 (46.9%)	
>5	79	43 (57.1%)	36 (42.9%)	0.167	35	17 (55.1%)	18 (44.9%)	0.112
T status								
T1/2	37	25 (54.2%)	12 (45.8%)		44	31 (50.0%)	13 (50.0%)	
T3/4	133	77 (54.1%)	56 (45.9%)	0.288	88	48 (55.4%)	40 (44.6%)	0.079
N status								
N0	58	43 (34.5%)	15 (65.5%)		61	43 (72.4%)	18 (27.6%)	
N1/2	112	59 (62.3%)	53 (37.7%)	0.007*	71	36 (46.4%)	35 (53.6%)	0.021*
Clinical stage								
I + II	69	50 (37.8%)	19 (62.2%)		70	49 (67.6%)	21 (32.4%)	
III	101	52 (63.9%)	49 (36.1%)	0.006*	62	30 (45.9%)	32 (54.1%)	0.011*

a Mean age. b Mean tumor size. *Statistically significant difference

In addition, eight fresh pairs of GC tissues and matched ANTs, were frozen and stored in liquid nitrogen until further use. A total of 20 pairs of primary and matched metastatic GC specimens were collected from archived paraffin-embedded tissues.

All the patients were followed up on regular basis and the Overall survival (OS) time was calculated from the date of surgery to the date of the death or when censured at the latest date if patients were still alive. Samples were obtained after given informed consent in accordance with the approval by institutional ethical review board.

### Cell culture

Five gastric cancer cell lines (AGS, BGC-823, HGC-27, MNK-28, MNK-45), and one immortalized human gastric epithelial mucosa cell line (GES-1) were obtained from the Cell Bank of the Chinese Academy of Sciences (Shanghai, China). All cell lines were grown in DMEM medium supplemented with 10% fetal bovine serum and 1% penicillin/streptomycin (Invitrogen).

### RNA isolation and quantitative real-time PCR

Total RNA was isolated using (Invitrogen, Calsbad, CA) from cultured cells and fresh tissues following the manufacturer’s instructions. Real-time PCR was performed on ABI7900HT Fast Real- Time PCR system (Applied Biosystems, Foster City, CA) system using SYBR Green SuperMix (Roche, Basel, Switzerland). Expression data were normalized to the Glyceraldehyde-3-phosphate dehydrogenase (GAPDH) or U6.

### Cell proliferation, wound-healing, migration and invasion assays

The CCK-8 assay was performed to test cell proliferation. Wound healing assays and transwell assays were performed to detect cell migration and invasion [11, 12]. The details were described in our previous study.

### Chromatin immunoprecipitation (ChIP), Western blotting analyses and immunofluorescence analyses

ChIP analysis, Western blotting analyses and immunofluorescence analyses were conducted according to the method described previously [11, 12]. The following antibodies were used in this study: C12orf59 (Novus), CDH11 (abcam), GAPDH (Cell Signaling Technology), E-cadherin (abcam), α-catenin (abcam), Vimentin (abcam), Fibronectin (abcam), NF-κB p65 (Cell Signaling Technology), p84 (Cell Signaling Technology), β-actin (R&D system), CXCR4 (abcam), FLT4 (Abnova), PTEN (Cell Signaling Technology) and TNFSF10(R&D system).

### Vector construction, transfection and retroviral infection

Plasmids encoding the human IκBα mutant (IκBα-mut) were gifts from Professor Song Libing (SYSUCC, Guangzhou, China). The following reagents were purchased from the GeneCopoeia Company (Guangzhou, China): CDH11 expression vector and its control vector; C12orf59 expression vector and its control vector; short hairpin RNA (shRNA) directed against C12orf5 and scrambled control; short interfering RNA (siRNA) specifically against p65 and scrambled control. Transfection was formed using Lipofectamine 2000 (Invitrogen) according to the manufacturer’s instructions. Cells transfected with empty vector were used as controls. The vectors were packaged into 293FT cells using the ViraPower Mix (Genecopoeia, Guangzhou, China). After 48 h’s culture, the lentiviral particles within the supernatant were harvested, filtered by centrifugation at 500 g for 10 min, and then transfected into GC cells.

### MiR-654-5p mimic, antagomir-654-5p, and transient transfection

The 3′-UTRs of C12orf59 were amplified and cloned downstream to the luciferase gene in a modified pGL3 control vector. MiR-654-5p mimic, antagomir-654-5p and their corresponding control oligonucleotides (Ribobio, GuangZhou, China) were transfected into GC cells cultured in six-well plates using Lipofectamine 2000 (Invitrogen) following the manufacturer’s instructions.

### Human umbilical vein endothelial cells (HUVEC) tube-formation assay

HUVECs were plated in a 24-well plate (5 × 103 per well) coated with Matrigel (BD Pharmingen, San Jose, CA, USA), and cultured at 37 °C in 5% CO2 for 24 h in the absence or presence of GC cell culture medium. The number of branch points of individual polygons of the capillary network was quantified in five low-power fields. Transwell assay was applied to examine the migration of HUVECs.

### Immunohistochemistry (IHC) staining assays and selecting the optimal cutoff value

The Dako Real Envision Kit (K5007, Dako) was used in IHC staining to visualize protein expression with primary antibody: C12orf59 (Novus) or CDH11 (abcam). Two independent, experienced pathologists evaluated and performed the IHC scoring as follows: The intensity of the staining was graded: 0 = no staining, 1 = weak staining, 2 = moderate staining, and 3 = strong staining. Tumor cells in five visual fields were randomly selected and scored on the basis of the percentage of positively stained cells (0–100%). The final IHC score was determined by multiplying the intensity score with the percentage of positive cells (range from 0 to 3).

To achieve the optimal cutoff value for C12orf59 IHC staining, we performed the X-tile plots analysis (Yale University School of Medicine, New Haven, CT, USA) [13]. At first, we used the X-tile program software to obtain the optimal C12orf59 IHC cutoff score to accurately classify patients according to clinical outcome in the training cohort. In the validation cohort, the cutoff score derived from X-tile analysis was investigated to test the association of C12orf59 expression with patients’ overall survival. X-title data were presented in a right triangular grid where each point represents a different cut point. The intensity of the color of each cutoff point represents the strength of the association. The X-tile program can automatically select the optimal data cut point according to the highest chi-square value (minimum *P*-value) defined by Kaplan–Meier survival analysis and log-rank test [14]. X-tile plots were performed with X-tile software version 3.6.1 (Yale University School of Medicine, New Haven, CT, USA).

### Cell fractionation assay

The cell fraction assay was carried out with the PARIS Kit (Life Technologies, Carlsbad, CA, USA) following the manufacturer’s instructions and p84 was used as positive control for nucleus and β-actin was used a positive control for cytoplasm.

### Experimental in vivo metastasis model

Six 4-week-old male BALB/c nude mice in each experimental group were injected with MKN-45/shC12orf59 or MKN-45/shcontrol, and HGC-27/C12orf59 or HGC-27/control cells, respectively. Briefly, 2*10^5^ cells were injected intravenously through tail vein into each mouse in a laminar flow cabinet. Six weeks later, mice were killed and examined. All the procedures were carried out in accordance with the guidelines of the Laboratory Animal Ethics Committee of Sun Yat-Sen University.

### Luciferase reporter assay

The wild type C12orf59 and CDH11 promoter and a promoter with mutated NF-κB-binding sites were constructed from Gene Copoeia company (Guangzhou, China), and the Cignal Finder 10-Pathway Reporter Array plates were purchased from QIAGEN company (Dusseldorf, GER). The reporter plasmids for detecting the transcriptional activity of NF-κB were generated as described previously [11]. The firefly luciferase construct was cotransfected with a control Renilla luciferase vector. Luciferase and renilla signals were measured 48 h after transfection using the Dual Luciferase Reporter Assay Kit (Promega Corporation), according to the manufacturer’s protocol.

### The cancer genome atlas (TCGA) data analysis

The Stomach Adenocarcinoma (STAD) patient clinical and RNA Sequencing data were downloaded from the Broad GDAC Firehose database (Broad Institute TCGA Genome Data Analysis Center (2016).

C12orf59 expression levels of STADs and normal tissues were compared by paired t-test, the two patient cohorts were compared using the Kaplan-Meier method, and the Cox proportional hazards model was used to compute the hazard ratio. *P* value of < 0.05 was considered statistically significant. For statistical assessments and plotting, R software version 3.4.3 (R Core Team (2017)) was used.

### Statistical analysis

Each experiment was repeated for three times or more. Statistical analysis was performed using an SPSS software package (SPSS Standard version 16.0, SPSS Inc) or GraphPad Prism 5.0. Comparisons between groups for statistical significance were analyzed with a two-tailed Student’s t test. Differences between variables were carried out using the Chi-square test or Fisher’s exact test. Survival analysis was performed using the Kaplan-Meier method and evaluated using the log-rank test. Multivariate survival analysis was assessed on all parameters that were found to be significant in univariate analysis using the Cox regression model. *P* values < 0.05 were considered significant.

## Results

### C12orf59 expression is increased and associated with poor outcome in GC

Consistent with the TCGA data analysis (Additional file 1: Figure S1a), we detected that the mRNA and protein level of C12orf59 was significantly up-regulated in 8 fresh GC tumor samples, compared with paired normal tissues. We also found that C12orf59 expression was higher in five GC cells than in GES-1 (Fig. 1a).

**Fig. 1:** C12orf59 is elevated in GC tissues and correlated with poor survival outcome in GC patients. **a** Left panel: Western blotting (upper) and qPCR (lower) analysis of C12orf59 protein expression in 8 pairs of matched GC tissues (T) and adjacent noncancerous tissues (ANT). Right panel: Western blotting (upper) and qPCR (lower) assay of C12orf59 expression in GSE1 and five GC cell lines; GAPDH was used as a loading control. **b** Representative image of negative C12orf59 IHC staining (Scoring intensity = 0) in normal gastric tissues, and representative images of negative Scoring intensity = 0), weak (Scoring intensity = 1), moderate (Scoring intensity = 2) and strong (Scoring intensity = 3) C12orf59 IHC staining in GC tissues is shown. **c** X-tile plots of the prognostic marker of C12orf59 in the two GC cohorts. X-tile analysis was carried out on patient data from the training cohort, equally subdivided into training and validation subsets. X-tile plots of training sets are displayed in the left panels, with matched validation sets in the smaller inset. The plot showed the χ2 log-rank values created when the cohort was divided into two populations. The cut point was demonstrated on a histogram of the entire cohort (middle panels) and a Kaplan–Meier plot (right panels). *P* values were defined by using the cut point derived from a training subset to parse a separate validation subset. (Upper panel) C12orf59 expression was divided at the optimal cut point, as defined by the most significant on the plot (with positive staining of C12orf59; *P* < 0.001). (Lowe panel) The optimal cut point for C12orf59 expression determined by X-tile plot of the testing cohort was applied to the validation cohort and reached high statistical significance (*P* < 0.001). The IHC score was determined by multiplying the intensity score with the percentage of positive cells in tumor tissues. **d.** IHC analysis of C12orf59 expression in primary and metastatic GC tissues. **e.** ROC curve analysis for different clinicopathological features and C12orf59 expression was performed to evaluate the survival status. Left panel: age (AUC = 0.575; *P* = 0.104), gender (AUC = 0.501; *P* = 0.975), grade (AUC = 0.393; *P* = 0.540), tumor size(AUC = 0.572; *P* = 0.119), T status (AUC = 0.631; *P* = 0.005), N status (AUC = 0.651; *P* = 0.001), clinical stage (AUC = 0.689; *P* < 0.001) and C12orf59 expression (AUC = 0.840; *P* < 0.001) implied statistical associations with survival in the training cohort; Right panel: age (AUC = 0.543; *P* = 0.443), gender (AUC = 0.538; *P* = 0.500), grade (AUC = 0.564; *P* = 0.257), tumor size(AUC = 0.604; *P* = 0.066), T status (AUC = 0.595; *P* = 0.092), N status (AUC = 0.665; *P* = 0.004), clinical stage (AUC = 0.693; *P* = 0.001) and C12orf59 expression (AUC = 0.663; *P* = 0.004) were used to test the survival status in validation cohort

To investigate the prognostic significance of in GC samples, we performed IHC staining for in two independent cohorts of GC samples. C12orf59 protein was stained in the cytoplasm, and significantly higher expressed in tumor tissues than in adjacent normal mucosal tissues (Fig. 1b). In the training cohort, the cutoff point (IHC score: 1.7) for dividing tumors into low- and high-expression of C12orf59 was determined using X-tile software. This optimal cut point determined by the training cohort was then applied to the validation cohort, which also identified high statistical significance again (*P* < 0.001; Fig. 1c). According to this cut point, high C12orf59 expression was observed in 102 of 170 (60.0%) GC samples in the training cohort (*P* < 0.001), and 79 of 132 (59.8%) GC samples in the validation cohort. This prognostic value for C12orf59 expression levels was also confirmed using a large cohort of 415 GC patients retrieved from the TCGA database (*P* = 0.017, hazard ratio (HR) = 1.59, 95% confidence interval (CI): (1.09–2.34), Additional file 1: Figure S1b).

In addition, high expression of C12orf59 was positively associated with N status (*P* = 0.007; *P* = 0.012, respectively) and overall clinical stage (*P* = 0.006; *P* = 0.011, respectively) both in training and validation cohorts of GC cases (Table 1), implying a potential role of C12orf59 in promoting GC metastasis. To investigate the role of C12orf59 in GC metastasis, C12orf59 expression was compared using IHC assay in 20 pairs of primary and metastatic GCs specimens. Overall, 18 pairs of GCs (90%) showed higher levels of C12orf59 expression in metastatic lesions, compared with the corresponding primary tumor samples (Fig. 1d).

Multivariate analysis showed that high expression of C12orf59 was an independent risk factor for adverse overall survival (OS) in both training (HR: 13.012; 95% CI: 6.402–26.446, *P* < 0.001; Table 2) and validation cohorts (HR: 2.656, 95% CI: 1.311–5.380, *P* = 0.007; Table 2). To further confirm the prognostic value of C12orf59 expression in GC, receiver operating characteristic (ROC) curves were plotted to test patient survival status. According to the ROC curve analysis, C12orf59 was found to be a promising predictor for survival status both in training (area under the curve (AUC) = 0.840; *P* < 0.001) and validation cohort (AUC = 0.663; *P* = 0.004; Fig. 1e).

**Table 2:** Univariate and Multivariate analysis of C12orf59 expression and various clinicopathological parameters in training and validation cohort patients with GC

Variables	Training cohort				Validation cohort			
	Case	HR	95% CI	*P*-value	Case	HR	95% CI	*P*-value
Univariate analysis								
Age								
≤ 60^a^	100	1.0			78	1.0		
>60	70	1.751	1.059–2.895	0.029	54	1.195	0.620–2.301	0.595
Gender								
Female	109	1.0			88	1.0		
Male	61	0.992	0.588–1.672	0.975	44	1.316	0.673–2.574	0.422
WHO grade								
G1/2	56	1.0			38	1.0		
G3	114	1.265	0.723–2.214	0.411	94	1.911	0.836–4.364	0.125
Tumor size(cm)								
≤ 5^b^	91	1.0			97	1.0		
>5	79	1.758	1.060–2.916	0.029*	35	2.165	1.116–4.203	0.022
T status								
T1/2	37	1.0			44	1.0		
T3/4	133	7.234	2.264–23.119	0.001*	88	2.304	1.008–5.264	0.048*
N status								
N0	58	1			61	1		
N1	112	3.722	1.833–7.558	< 0.001	71	3.823	1.738–8.409	0.001*
Clinical stage								
I + II	69	1			70	1		
III	101	4.677	2.371–9.227	< 0.001	62	4.308	2.022–9.180	< 0.001*
C12orf59 expression								
Low expression	102	1.0			79	1.0		
High expression	68	13.497	6.790–26.832	< 0.001*	53	3.326	1.680–6.582	0.001*
Multivariate analysis								
Age								
≤ 60^a^	100	1.0			78	1.0		
>60	70	0.98	0.580–1.657	0.941	54	1.021	0.520–2.007	0.952
T status								
T1/2	37	1.0			44	1.0		
T3/4	133	6.351	1.944–20.752	0.002	88	1.35	0.568–3.210	0.497
N status								
N0	58	1.0			61	1.0		
N1	112	1.690	0.818–3.489	0.156	71	2.875	1.269–6.512	0.011*
Tumor size(cm)								
≤ 5^b^	91	1.0			97	1.0		
>5	79	1.405	0.832–2.374	0.203	35	1.404	0.701–2.810	0.338
C12orf59 expression								
Low expression	102	1.0			79	1.0		
High expression	68	13.012	6.402–26.446	< 0.001*	53	2.656	1.311–5.380	0.007*

a Mean age. b Mean tumor size. Cox propotional hazard regression model, enter; *HR* Hazard ratio, *CI* Confidence interval;*Statistically significant difference

### C12orf59 promotes GC invasion and metastasis

To explore the oncogenic role of C12orf59 in GC, we suppressed C12orf59 expression in MKN-45 and AGS cell lines that have high levels of C12orf59, and overexpressed C12orf59 expression in HGC-27 cell lines that have low level of C12orf59 (Fig. 2a). We found that C12orf59 knockdown did not influence cell proliferation (Additional file 2: Figure S2). However, suppression of C12orf59 significantly inhibited the ability of MKN-45 and AGS cells to fill the wound gap (Fig. 2b) and migrate through Transwell membranes (Fig. 2d). Also, C12orf59 inhibition largely reduced GC cell invasive ability, as measured by Boyden chamber assays (Fig. 2d). On the other side, enforced overexpression of C12orf59 in HGC-27 cells substantially increased cell migration and invasive capacity (Fig. 2c and e).

**Fig. 2:** The expression levels of C12orf59 influence the aggressive capacity in vitro and metastasis in vivo. **a** Western blotting shows that the levels of C12orf59 were largely decreased by the treatment with C12orf59-shRNA-1 or C12orf59-shRNA-2 in MKN-45 and AGS cells, while potentially increased in HGC-27/C12orf59 cell line. **b** C12orf59 deletion dramatically reduced the migratory ability of GC cells in a wound-healing assay. **c** Wound-healing assays demonstrate that HGC-27/C12orf59 cells had higher motility than that in HGC-27/vector cells. **d** Downregulation of C12orf59 resulted in a decrease in the migratory and invasive abilities of GC cells as determined by Transwell analysis. **e** Overexpression of C12orf59 in HGC-27 cells increased their migratory and invasive abilities. **f** Representative hematoxylin and eosin (H&E) staining depicting metastatic tumors in the lung of nude mice that originated from MKN-45/shC12orf59 and MKN-45/shcontrol cells injected via the tail vein (left). Number of metastatic nodules formed in the lung of mice 6 weeks after tail vein injection of MKN-45/shC12orf59 or MKN-45/shcontrol cells. Six mice per group; *P < 0.01. **g** H&E staining depicting metastatic tumors in the lung of nude mice that originated from HGC-27/vector and HGC-27/C12orf59 cells injected via the tail vein (left). Number of metastatic nodules formed in the lung of mice 6 weeks after tail vein injection of HGC-27/vector or HGC-27/C12orf59 cells. Six mice per group; *P < 0.01

To further validate the effect of C12orf59 on tumor metastasis, in vivo metastasis assay was performed in nude mice: MKN-45/shC12orf59 or MKN-45/shcontrol, and HGC-27/C12orf59 or HGC-27/control cells were injected into nude mice via tail vein, respectively. In accordance with previous results, the mice injected with MKN-45/shC12orf59 cells formed fewer nodes per lung compared with the shcontrol group (2.2 ± 1.7 versus 7.0 ± 2.8, *P* < 0.001), while the mice injected with HGC-27/c12orf59 formed more nodes per lung compared with the control group (6.5 ± 2.4 versus 2.7 ± 1.2, *P* < 0.001). Histological studies confirmed that the lesions were caused by extravasation and subsequent tumor growth of GC cells into the lungs (Fig. 2f and g).

### C12orf59 induces epithelial-mesenchymal transition (EMT) and promotes angiogenesis in GC

EMT plays an important role in tumor invasion and metastasis [15, 16]. In our study, we observed that overexpression of C12orf59 in HGC-27 cells markedly enhanced the levels of the mesenchymal marker Vimentin and Fibronectin, and concomitantly reduced the expression of the epithelial markers E-cadherin and α-catenin. Opposite expression patterns of these genes were observed in C12orf59 knockdown cells (Fig. 3a). Immunofluorescence staining confirmed the down-regulated expression of E-cadherin and the up-regulated expression of Vimentin in C12orf59-transfected cells (Fig. 3b). Angiogenesis is a key step in the cancer invasion-metastasis cascade [17], thus we also explored whether C12orf59 is likely to be involved in GC angiogenesis using an in vitro human umbilical vein endothelial cell (HUVEC) model. We observed that overexpressing C12orf59 potently enhanced, while silencing C12orf59 strongly inhibited, the ability of GC cells to induce tube formation and migration of HUVECs (Fig. 3c and d). In addition, the microvessel density (MVD) (as indicated by anti-CD31 staining) was significantly stronger in GC samples with C12or59 high expression than GC samples with C12orf59 low expression in the training cohort of 170 samples (Additional file 3: Figure S3).

**Fig. 3:** Expression level of C12orf59 influence GC EMT and angiogenesis. **a** Western blotting reveals that knockdown of C12orf59 by shRNAs resulted in an increased expression of E-cadherin and α-catenin and a decreased expression of fibronectin and vimentin in both MKN-45 and AGS cells, compared with that in shcontrol treated cells. Decreased levels of E-cadherin and α-catenin and increased levels of fibronectin and vimentin were examined in HGC-27/C12orf59 cells compared with that in control HGC-27/vector cells. **b** IF staining shows a downregulated expression of E-cadherin and an upregulated expression of vimentin in HGC-27/C12orf59 cells compared with that in control HGC-27/vector cells with a corresponding change in the number of positive staining cells. **c** and **d.** The abilities of in vitro capillary tube formation (**c**) and migration (**d**) of HUVEC were significantly decreased after incubating with culture medium of C12orf59-silenced GC cell, while potentially strengthened after incubating with culture medium of C12orf59-transfected GC cell

### C12orf59 promotes GC cells’ migration and invasion abilities by enhancing CDH11 expression

To further determine the potential downstream targets regulated by C12orf59 in promoting GC cells invasion and/or metastasis, mRNA expression profiles of MKN-45/shC12orf59 cells were compared with that of control MKN-45/shControl cells using a Human Tumor Metastasis RT^2^ Profiler PCR Array containing 84 cell metastasis-related genes. As shown in Fig. 4a, three downregulated genes (that is, CDH11, CXCR4 and FLT4) and two upregulated genes (that is, PTEN and TNFSF10), showed a more than twofold change in mRNA levels in MKN-45/shC12orf59 cells compared with that in MKN-45/shControl cells (Additional file 4: Table S1). Subsequently, we validated that two targets CDH11 and CXCR4 were up-regulated in protein level by western blot assay in cell after C12orf59 knockdown, but the other genes did not exhibit differential protein expression before and after depletion of C12orf59 (Fig. 4b). In addition, a significant positive correlation between the expression of C12orf59 and CDH11 was evaluated in our cohort of GC tissues (Fig. 4c, *P* < 0.05). However, we did not observe significant correlation between CXCR4 and CDH11in high and low expression groups.

**Fig. 4:** CDH11 is responsible for C12orf59-induced GC cell invasiveness and EMT. **a** The five genes, CDH11, CXCR6, FLT4, PTEN, and TNFSF10, were examined 2-fold mRNA differential expression in MKN-45/shC12orf59 cells compared with that in MKN-45/shControl cells by using a Human Tumor Metastasis RT2 Profiler PCR Array. **b** Silence of C12orf59 by shRNA in MKN-45 cells substantially downregulated CDH11 and CXCR4 expression as examined by western blotting. **c** The expression level of C12orf59 and CDH11 were positively correlated in the training cohort of 170 GC samples examined. **d** Wound-healing assays showed that CDH11 overexpression increased the migratory ability of C12orf59-depleted MKN-45 cells. **e** Transwell analysis indicated that CDH11 overexpression enhanced the migratory and invasive abilities of C12orf59-depleted MKN-45 cells. **f** Western blotting shows that after restoration of CDH11 in MKN-45/ shC12orf59 cells, the levels of E-cadherin and α-catenin decreased, whereas the levels of fibronectin and vimentin increased. **g** IF staining demonstrates a downregulated expression of E-cadherin and an upregulated expression of vimentin in MKN-45/shC12orf59 cells, after overexpression of CDH11. **h and i.** Restoration of CDH11 antagonized the inhibitory effects of C12orf59 knockdown on the abilities of capillary tube formation (**h**) and in vitro migration (**i**) of HUVECs

Next, we try to explore whether CDH11 is involved in C12orf59-induced GC cell invasiveness and EMT. Wound-healing and Transwell assays showed that after CDH11 was introduced, the compromised migrative and invasive capacities of C12orf59-silenced MKN-45 cells were all largely restored (Fig. 4d and e). And meanwhile, we observed the decreased expression of epithelial markers (E-cadherin and α-catenin) and increased expression of mesenchymal markers (fibronectin and vimentin) after overexpression of CDH11 in C12orf59-silenced cells (Fig. 4f). IF staining of E-cadherin and vimentin also confirmed this result (Fig. 4g). In addition, the tube formation and migration of HUVECs were also largely strengthened when CDH11 was restored in C12orf59-silenced cells (Fig. 4h and i). The in vivo metastasis ability assay also showed that after re-introduction CDH11 in MKN-45/shC12orf59 cells, the in vivo metastasis ability was largely enhanced (Additional file 5: Figure S4).

### C12orf59 promotes CDH11 expression via NF-κB dependent transcription

To identify the potential downstream pathway modulated by C12orf59, we performed luciferase experiments using the Cignal Finder 10 Pathway Reporter Arrays and Dual-Glo Luciferase Assay System. Among the ten different pathways, transcriptional activity of NF-κB pathway was compromised predominantly when C12orf59 was overexpressed (Fig. 5a). This phenomenon promoted us to exam the effluence of C12orf59 on NF-κB in GC cells. We further confirmed that, the stimulatory effect of C12orf59 on NF- κB activation was dramatically inhibited upon IκBα-mut (IκBα-dominant-negative mutant, which is widely known to inhibit the NF-κB pathway) transfection (Fig. 5a). Moreover, subcellular fraction assays showed overexpressing C12orf59 led to stronger nuclear localization of NF-κB p65 (Fig. 5b). Collectively, these results suggest that C12orf59 plays an important role in regulation of NF-κB signaling in gastric cancer.

**Fig. 5:** C12orf59 activates CDH11 expression through NF-κB signaling. **a** Luciferase reporter assay was performed in C12orf59 overexpressed GC cells and control cells, respectively (right). Remarkable activation of NF-κB signaling pathway is observed after C12orf59 was overexpressed. **b** Western blotting showed increased expression level of nuclear NF-κB p65 after overexpression of C12orf59 in GC cells. **c** Schematic illustration of CDH11 promoter. One potential NF-κB p65 binding sites was shown. **d** ChIP assay showed the binding to NF-κB p65 to CDH11 promoter in vivo. The promoter region of CDH11 was amplified from the DNA recovered from the immunoprecipitation complex using a specific antibody for p65. The following PCR primers for ChIP assays were used: 5′- GTCCTTGGCGTGATTCCTAA-3′, 5′- TACGGGAGAAAGGGCCTAAT-3′. **e** Luciferase reporter assay of CDH11 promoter showed remarkable activation is observed when C12orf59 was overexpressed. **f** Western blotting showed decreased expression level of CDH11 after transfection of sip65 in HGC-27/C12orf59 cells. **g** Wound-healing assays showed that sip65 transfection inhibited the migratory ability of C12orf59-overexpressing HGC-27 cell. **h** Transwell analysis indicated that enhanced the migratory and invasive abilities of C12orf59-overexpressing HGC-27 cell were largely compromised after treatment with sip65. **i** Western blotting shows that after sip65 transfection in HGC-27/C12orf59 cells, the levels of E-cadherin and α-catenin increased, whereas the levels of fibronectin and vimentin decreased. **j** IF staining demonstrates an upregulated expression of E-cadherin and a downregulated expression of vimentin in HGC-27/C12orf59 cells, after treatment with sip65. **k** and **l.** sip65 transfection largely attenuate the enhanced effects of C12orf59 overexpression on the abilities of capillary tube formation (**k**) and in vitro migration (**l**) of HUVECs

As NF-κB could activate transcription of specific genes and was involved in C12orf59-mediated GC pathogenesis, we thus try to investigate if C12orf59 upregulated CDH11 expression is mediated by NF-κB in GC cells. We analyzed CDH11’s promoter sequence using the PROMO algorithm and identified one putative NF-κB p65-binding site inside the putative CDH11 promoter region (Fig. 5c). As anticipated, the chromatin immunoprecipitation results showed that the enrichment of NF-κB p65 on the promoter of CDH11 was substantially enhanced in HGC-27/C12orf59 cell line. On the other hand, after knockdown of p65 by siRNA in HGC-27 cells, the enrichment of NF-κB on the CDH11 promoter was substantially reduced (Fig. 5d). Next, we cloned the putative CDH11 promoter sequence into a pGL4-basic vector, and transfected into GC cell. The dual luciferase reporter assay showed that overexpression of C12orf59 dramatically enhanced the transcription activity of firefly luciferase. However, when the binding sequence was deleted, the firefly luciferase expression dropped significantly (Fig. 5e). Further functional studies showed that C12orf59-mediated enhanced CDH11 expression, migrative/invasive capacity, EMT and angiogenesis ability of HGC-27/C12orf59 cells were all prevented, when NF-κB p65 was inhibited (Fig. 5f, g, h, i, j, k and l).

### Bidirectional regulation between C12orf59 and CDH11 via NF-κB in GC

To identify the upregulation mechanism of C12orf59 in GC, we performed In silico analysis, and detected that C12orf59 promoter contained putative NF-κB p65 binding sites (Fig. 6a). Additional study detected that overexpression of CDH11 in GC could enhance NF-κB-induced luciferase activity, and promote nuclear localization of NF-κB p65, suggesting CDH11 is a positive regulator of NF-κB signaling (Additional file 6: Figure S5). Thus, we tried to explore weather CDH11 could in turn up-regulate C12orf59 expression via NF-κB. The chromatin immunoprecipitation results showed that after overexpression of CDH11, more p65 proteins were recruited to the binding sites in C12orf59 promoter. When NF-κB p65 was inhibited by siRNA, the enrichment of p65 protein on C12orf59 promoter was significantly decreased (Fig. 6b). The dual-luciferase reporter assay revealed that ectopic expression of CDH11 activated the transcription of firefly luciferase that was driven by the wide-type C12orf59 promoter. When the binding sequence was deleted, firefly luciferase expression dropped dramatically (Fig. 6c). Furthermore, we observed that overexpression of CDH11 increased C12orf59 mRNA and protein levels in GC cells. On the other hand, C12orf59 levels were decreased when NF-κB p65 was inhibited (Fig. 6d). Thus, CDH11 could in turn enhance C12orf59 expression via NF-κB, and thus form a positive feedback loop, which sustained the metastatic and aggressive phenotype of human GC cells (Fig. 6e).

**Fig. 6:** Bidirectional regulation between CDH11 and C12orf59. **a** Schematic illustration of C12orf59 promoter. One potential NF-κB p65 binding sites was shown. **b** ChIP analysis of NF-κB p65 binding on C12orf59 promoter. ChIP DNA was quantified by real-time PCR primers specific to human C12orf59 promoter. The following PCR primers for ChIP assays were used: 5′- GGAGATCGAGACCATTCTGG-3′, 5′- AAACTCTGCCTCCTGGGTTC-3′. **c** Fragments encompassing the putative C12orf59 promoter region were inserted upstream of firefly luciferase coding sequences in the pGL3-basic plasmid. The effect of NF-κB protein on transcriptional activity of C12orf59 promoter was measured by luciferase reporter assays. **d** Overexpression of CDH11 increased C12orf59 mRNA and protein level, while inhibition of NF-κB p65 decreased C12orf59 mRNA and protein level in GC cells. **e** Molecular mechanism of the C12orf59/ NF-κB/CDH11 feedback loop in promoting GC metastasis

### C12orf59 is negatively regulated by miR-654-5p

It is known that post-translational regulation such as microRNA (miRNA) might play critical roles in protein regulation, thus we investigate the potential miRNA regulators of C12orf59 in GC. We performed bioinformatics analyses(TARGETSCAN) and overlapped the predicted miRNA regulators with the downregulated miRNAs from miRNA expression profiles of GC [18]. The result showed that miR-654-5p was singled out as a potential regulator of C12orf59 (Fig. 7a). Our qRT-PCR analysis showed that miR-654-5p was indeed downregulated in GC tissues and cell lines examined (Fig. 7b). In addition, overexpression of miR-654-5p decreased the luciferase activity of C12orf59 3′-UTR (Fig. 7c). Meanwhile, the C12orf59 mRNA and protein levels were all substantially reduced after overexpression of miR-654-5p in GC cells (Fig. 7d and e). However, miR-654-5p-mut failed to exert none of the above effects. These data suggested miR-654-5p directly suppress C12orf59 expression and decreased miR-654-5p might contribute to C12orf59 overexpression in GC at least partially. At last, we examined investigate the phenotypes of miR-654-5p in GC cells. After overexpression of miR-654-5p in GC cell, we detected that the invasion and metastatic ability was largely compromised (Additional file 7: Figure S6).

**Fig. 7:** MiR-654-5p is a negative regulator of C12orf59. **a** Illustration of screening miRNAs regulating C12orf59: Method #1 used the prediction algorithm of TARGETSCAN identified miRNAs, which hold potential as C12orf59 suppressors. Method #2 used miRNA profiling and identified miRNAs, which were downregulated significantly in GC. Then, we overlapped the results of two methods and singled out miR-654-5p as a potential regulator. **b** Quantitative RT-PCR assay of miR-654-5p expression in six GC cell lines (left panel), and in eight pairs of matched GC (T) and adjacent non-neoplastic gastric tissue (ANT) (right panel). **c** Predicted miR-654-5p target sequence in 3′-UTR of C12orf59 (C12orf59 3′-UTR) and mutant miRNA containing three altered nucleotides in the seed sequence of miR-654-5p (miR-654-5p-mut). **d** Luciferase assay of pGL3- C12orf59 3′-UTR reporters co-transfected with increasing amounts (10, 20 and 50 nM) of miR-654-5p mimic or miR-654-5p-mut in MNK-45 and AGS cell lines. **e** Western blotting analysis demonstrates that miR-654-5p transfection markedly decreased C12orf59 protein levels of MNK-45 and AGS cells, whereas miR-654-5p-mut exerted no inhibition effect. *P < 0.05

## Discussion

In the present study, we identified the putative oncogene, *C12orf59*, is frequently overexpressed in GC cell lines and tissues. More importantly, high *C12orf59* expression was associated with malignant clinicopathological characteristics and poor survival outcome in two independent cohorts of GC samples. Thus, the examination of C12orf59 expression by IHC could be used as an additional tool in distinguishing GC patients at high risk of metastasis and/or progression, which might provide some useful information for clinicians in optimizing individual therapy management for GC disease. As a newly identified gene, the expression pattern and clinical feature of *C12orf59 i*n human cancers is largely unknown. In contrast to our finding, Xie reported the loss of *C12orf59* expression is a common feature of Renal cell carcinoma that is correlated with increased aggressive tumor behavior and predicts poor survival outcomes of patients, suggesting a potential tumor-suppresive role of *C12orf59* in this disease [10]. These results, collectively, suggested that the biologic/clinical significance of *C12orf59* expression in different human cancers may be tissue-specific. Clearly, further investigations are substantially needed to identify the expression dynamics of *C12orf59* and its clinicopathological/prognostic significance in other human cancer types.

Based on the clinical finding, we carried out a series of in vitro and in vivo experiments to explore the potential mechanisms. Our results show that enforced knockdown or ectopic overexpression of *C12orf59* in GC cells substantially repressed or promoted the capacities of invasion, migration, and EMT, respectively. In an experimental in vivo metastasis model, we further noticed that the tail injection of ectopic overexpression of C12orf59 in GC cells led to a significant increase in the number of lung metastatic lesions. These data supported strongly the view that C12orf59 has a crucial oncogenic role in the promotion of GC cells invasive and/or metastatic process, and C12orf59 could provide an attractive potential target for the development of novel therapeutic interventions in GC.

To gain a further insight into the downstream molecular events involving *C12orf59* and GC invasiveness and/or metastasis, we used a Human Tumor Metastasis RT^2^ Profiler PCR Array containing 84 cell metastasis-related genes was used to compare mRNA expression profiles between MKN-45/shControl cells and MKN-45/shC12orf59 cells. We found and validated that CDH11 was the downstream target of C12orf59 in GC cells. To date, the gene functions of CDH11 in human cancers are complicated and it exhibited distant role in different tumor types. The CDH11 functioned as an oncogene in certain human cancers, such as breast, pancreatic, colorectal and prostate cancers [19–23]. In glioma, osterosarcoma and cervical cancer, however, it was reported to exert tumor-suppressor functions [24–27]. Up to date, however, the expression pattern and potential biological function of CDH11 in human GC have not been elucidated. Our finding, for the first time, reported that C12orf59 enhances the binding of NF-κB to the promoter of CDH11, thereby promoting the aggressive phenotype of GC cells. Moreover, our study also found that CDH11 overexpression could in turn enhance C12orf59 expression via NF-κB. Thus, the bidirectional regulation of C12orf59 and CDH11 forms a positive feedback to promote the progression of GC cells. Previous studies have shown that positive feedback regulatory network could to form a self-sustained mode which is autonomous to the original stimuli [28–30]. Thus, we speculate that, once induced by NF-κB, the C12orf59/NF-κB/CDH11 feedback loop allows GC cells to become more autonomous, which could endow GC cells with more aggressive and invasive phenotype (Fig. 6e).

## Conclusion

In summary, our current report describes, for the first time, the important oncogenic role of C12orf59 in GC metastasis. Functional and mechanistic investigations showed that C12orf59 promoted GC metastasis and invasion by up-regulating CDH11 through NF-κB. Interestingly, up-regulated CDH11 could in turn enhance C12orf59 expression via NF-κB, which form a positive feedback loop, and thus sustained the metastatic and aggressive nature of human GC cells. Therefore, targeting C12orf59/NF-κB/CDH11 loop may represent a new therapeutic strategy to improve treatment and survival of GC patients.

## Additional files

Additional file 1: **Figure S1.** TCGA data analysis of C12orf59 expression pattern and prognostic value in GC tissues. **a.** Expression of C12orf59 mRNA level in 68 paired GC and adjacent normal tissues from TCGA database. The mean level of C12orf59 expression in the GC tissues was significantly higher than in normal tissues (*P < 0.001, paired t-test). **b.** High expression of C12orf59 in GC is correlated with poor overall survival in the TCGA gastric cancer data set. Kaplan-Meier analysis of overall survival (OS)of patients with GC for whom OS information was available in TCGA the Stomach Adenocarcinoma (STAD) data set. C12orf59-low and C12orf59-high are defined by the median value of C12orf59 expression. (DOCX 149 kb)

Additional file 2: **Figure S2.** Suppression or overexpression of C12orf59 did not alter the GC cellular growth rate. (DOCX 155 kb)

Additional file 3: **Figure S3.** The microvessel density (MVD), as indicated by CD31 staining was noticeably stronger in GC samples with C12orf59 high expression compared with GC samples with C12orf59 low expression in the training cohort of 170 samples. *P < 0.05. (DOCX 108 kb)

Additional file 4: **Table S1.** List of genes differentially expressed in MKN-45 cells after C12orf59 knockdown using a Human Tumor Metastasis Real-time PCR Array. (DOCX 24 kb)

Additional file 5: **Figure S4.** Restoration of CDH11 in GC cells enhanced the in vivo metastasis ability. Representative hematoxylin and eosin (H&E) staining depicting metastatic tumors in the lung of nude mice that originated from MKN-45/shC12orf59/CDH11 and MKN-45/shC12orf59/control cells injected via the tail vein (left). Number of metastatic nodules formed in the lung of mice 6 weeks after tail vein injection of MKN-45/shC12orf59/CDH11 or MKN-45/shC12orf59/control cells. Six mice per group; **P < 0.01. (DOCX 156 kb)

Additional file 6: **Figure S5.** CDH11 activates NF-κB signaling**. a.** Luciferase reporter assay showed NF-κB signaling pathway is activated after CDH11 was overexpressed. **b.** Western blotting showed increased expression level of nuclear NF-κB p65 after overexpression of CDH11 in GC cells. (DOCX 120 kb)

Additional file 7: **Figure S6.** miR-654-5p inhibited GC cell invasion and metastatic ability in vitro*.* **a.** Overexpression of miR-654-5p dramatically reduced the migratory ability of GC cells in the wound-healing assay. **b.** Overexpression of miR-654-5p resulted in a decrease in the migratory and invasive abilities of GC cells as determined by Transwell analysis. *P < 0.05. (DOCX 141 kb)

## Abbreviations

AUC: Area under the curve
C12orf59: Chromosome 12 open reading frame 59
ChIP: Chromatin immunoprecipitation
CI: Confidence interval
EMT: Epithelial-mesenchymal transition
GC: Gastric cancer
HR: Hazard ratio
OS: Overall survival
ROC: Receiver operating characteristic
TCGA: The Cancer Genome Atlas
